# Brain Metastasis of Nasopharyngeal Carcinoma: A Case Report and Literature Review

**DOI:** 10.1155/2012/405917

**Published:** 2012-02-20

**Authors:** Orit Kaidar-Person, Jonathan Kuten, Fadi Atrash, Salem Billan, Abraham Kuten

**Affiliations:** Oncology Institute, Rambam Health Care Campus, P.O. Box 9602, Haifa 31096, Israel

## Abstract

Central nervous system metastases from nasopharyngeal carcinoma (NPC) are uncommon. The patient presented was diagnosed with aggressive advanced NPC resistant to treatment and complicated by a solitary brain metastasis. A PubMed database search was conducted to review the existing literature regarding brain metastases of NPC, using the search terms “nasopharyngeal neoplasia,” “nasopharyngeal carcinoma,” “nasopharynx,” “radiotherapy,” “central nervous system,” and “brain” in section of “Title/Abstract.” The articles were first evaluated by title and then by abstract, and thereafter appropriate manuscripts were evaluated by full text. References of the published papers were also reviewed.

## 1. Introduction

Nasopharyngeal carcinoma (NPC) is a rare malignancy with an incidence of 0.5–2 per 100,000 in Europe and the United States [1]. In certain places such as southern China and southeast Asia, the incidence rises significantly and these areas are considered endemic for NPC. Intermediate incidence rates are found in the Mediterranean Basin and the Arctic [1–3]. In Malaysia, NPC is the most common head and neck cancer and is second only to lung cancer among men [4].

 It is imperative to remember that although squamous cell carcinoma is the most common histological subtype of nasopharynx malignancy, it differs from other head and neck squamous cell carcinomas in epidemiology, etiology, histology, natural history, and response to treatment [1–4]. Etiology is multifactorially influenced by host of viral, genetic, and environmental contributors [5]. Epstein-Barr virus (EBV) infection was found to be a major contributor in the pathogenesis of NPC in both endemic and nonendemic areas and is ubiquitous in NPC, as the malignant cells contain multiple copies of the EBV genome regardless of histology or differentiation [5].

Symptoms of NPC can be obscure due to its anatomic location which begins in upper part of the pharynx behind the nose and ends at the proximal part of the trachea and esophagus. These include nasal, aural, and neurologic symptoms, thus often a challenge in diagnosis. Cervical lymphadenopathy is commonly noted in physical examination as the majority of newly diagnosed NPC patients have locoregionally advanced disease, and cervical nodes are usually involved [5]. More than 13% of the patients are presented with occult primary tumors.

 Treatment is usually composed of a nonsurgical approach as the anatomic location is difficult to manage and in most cases there is a locoregional disease; therefore, currently the standard of care for these patients consists of concurrent chemoradiotherapy with cisplatin-based regimens, generally followed by adjuvant chemotherapy [5]. This treatment approach results in cure for the vast majority of patients, with 3-year disease-free and overall survival rates of approximately 70% and 80%, respectively. Surgery is usually reserved for persistent or recurrent disease [5].

It is widely known that, although NPC can directly invade the skull base, true brain metastases of NPC are rare. The most common sites for distant NPC metastases are the bone, lung, and liver. A PubMed database search of existing English literature regarding brain metastases of NPC revealed few well-described cases. Other reports of central nervous system (CNS) involvement describe spinal or pituitary metastases. A case of aggressive NPC with a solitary brain metastasis and related literature is discussed.

## 2. Case Report

A 54-year-old male patient, Jewish Caucasian Israeli of North African descent, no history of chronic disease, no history of ethanol abuse or smoking. For 6 months prior to being diagnosed, the patient complained of tinnitus of left ear and hearing loss. The patient was referred by his family doctor to brain CT scan, which revealed an asymmetry at the left nasopharynx and no evidence of brain lesion. ENT evaluation included fiberoptic endoscopy, which indicated a bulb in the left nasopharynx. Biopsy was positive for poorly differentiated nasopharyngeal carcinoma. Fluorodeoxyglucose positron emission computed tomography (FDG-PET/CT) scan prior to treatment showed pathological uptakes at the left nasopharynx and left level II lymph nodes. Brain and cervical MRI did not show any skull base involvement or brain metastases. The patient was diagnosed with T3N1M0 (AJCC, 7th edition) poorly differentiated NPC. Thereafter, he received one cycle of induction chemotherapy (according to our department protocol) with cisplatin (100 mg/m^2^, day 1) and 5-fluorouracil (1000 mg/m^2^, days 1–5). The fifth day of 5-fluorouracil was omitted due to acute renal failure, which resolved with conservative treatment. One month later, chemoradiotherapy was initiated using intensity-modulated radiation therapy: a total dose of 70 Gy to the tumor site and involved lymph node and 50 Gy to bilateral neck fields (all levels, excluding level Ia), concomitant with weekly carboplatin (area under the curve (AUC) of 2). FDG-PET/CT scan performed three months after completion of chemo-radiotherapy showed pathological uptakes in the left cervical lymph nodes and several uptakes in the lung that were suspicious for metastases. A biopsy taken from a lung lesion was positive for metastatic NPC. Chemotherapy regimen of carboplatin (AUC 6) and paclitaxel was introduced; however, radiological evaluation after three chemotherapy cycles indicated tumor progression, and treatment was changed to gemcitabine (single agent). Total body CT scan performed after three cycles of gemcitabine revealed progressive disease in the neck and lung and an occipital hypodense lesion suspicious for metastasis, which was not evident on a prior brain CT. Brain MRI excluded any additional brain lesions or direct tumor invasion to the brain (Figure 1). Biopsy from the brain lesion indicated positive staining for *in situ* hybridization for Epstein-Barr virus (EBV), while staining for TTF1 and P63 was negative. These results were consistent with NPC metastasis. The patient received a total radiation dose of 40 Gy (26.6 Gy per fraction) to the solitary brain lesion using volumetric modulated arc therapy (VMAT). Nonetheless, soon after completion of radiotherapy, the patient's performance status continued to deteriorate due to his systemic disease and he was offered best supportive care.

## 3. Discussion

Despite the fact that NPC has a distinctive ethnic and geographic distribution, immigration is a common phenomenon, and in some cases the incidence may still be high in immigrants and offspring [1–6].

The patient presented here, a male of North African descent, was diagnosed with extremely aggressive disease, including brain metastasis. Israel is considered to be a low-to-intermediate incidence area of NPC; however, the incidence in North Africa is relatively higher [1, 2]. Migrant epidemiological data showed that, even after immigration to Israel, the high incidence of NPC persisted among North African immigrants and their offspring, compared to the local population [1]. These results, among others, suggest that both genetic and environmental factors play an important role in the pathogenesis of NPC. This may also explain the fact that only a minor proportion of people infected with EBV developed NPC. Most patients diagnosed with NPC in Israel are found to have either nonkeratinizing carcinoma or undifferentiated carcinoma and are diagnosed at an advanced stage; both histology types are strongly associated with EBV [2, 3].

Brain metastases of NPC are rare. A PubMed database search revealed only a few well-described relevant cases. Other reports of CNS involvement describe spinal or pituitary metastases. This paper does not encompass reports of spinal involvement, leptomeningeal spread, or direct intracranial invasion. All the reports of brain metastases are summarized in Table 1 [7–12]. Every patient whose clinical information was reported had node-positive disease. Some reports did not indicate which radiological evaluation was undertaken to exclude direct invasion to the brain.

Liaw et al. [9] published an analysis of 352 cases of NPC to determine the pattern of distant metastases; of these, three were cases of CNS metastases, but no information was given regarding whether these represent cases with a single brain metastasis, the treatment these patients received, or their outcomes. Kuten et al. [7] reported a case of left occipital lobe NPC metastasis that presented 58 months from the end of the primary radiotherapy. In this case, in view of locally advanced disease at presentation, the patient received induction chemotherapy consisting of four drugs. Partial remission of the neck lymph nodes and the primary NPC site was attained prior to definitive radiotherapy. Total radiotherapy dose to the primary site was 62 Gy, with 60 Gy to the neck; a supplemented boost was given to involved sites, but the boost dose was not reported. Complete remission was achieved, and the patient remained well for 45 months.

The patient presented in this paper had an aggressive disease and progressed early after definitive radiotherapy, as noted by pathology-proven lung metastases.

Functional imaging is still under investigation in NPC; however, some reports suggested that a high standardized uptake value (SUV) on FDG-PET/CT scans has a potential value as a prognostic indicator. High pretreatment SUV had a significantly lower 3-year disease-free survival than patients with lower FDG uptake [13]. The patient present in this case had evidence of advance disease in FDG-PET/CT and relatively high pretreatment SUV count. FDG-PET/CT scan performed three months after completion of chemo-radiotherapy showed pathological uptakes in the left cervical lymph nodes with an SUV of 5 (Figure 2); however, there is no concrete evidence in regard to the value of posttreatment SUV as an indicator for survival [5, 13].

Kuten et al. [7] also reported that their patient had lung metastasis preceding the metastasis to the brain and, as in the presented case, EBV staining using *in situ* hybridization was positive. Their patient was treated with surgery and chemotherapy for both metastasis sites but died six months later due to the progressive metastatic lung disease. As evidenced by both these cases, the extent and control of the systemic disease are crucial in determining the prognosis after successful treatment of brain metastases. In the presented case, VMAT was applied for radiation of the brain lesion after brain MRI confirmed a solitary lesion. This technique combines 3D volumetric imaging and advanced treatment planning, thereby maximizing the radiation dose to the target and minimizing exposure to surrounding healthy tissues.

Another case of NPC occipital lobe metastases was reported by Ngan et al. [8]. In this case the patient had bilateral occipital lobe involvement diagnosed at presentation of NPC. The patient also had blastic bone lesions assumed to be of NPC origin after other malignancies were excluded, including prostate cancer. Biopsy of the brain lesion indicated squamous cell carcinoma; EBV status was not reported. The patient was treated with systemic chemotherapy and head and neck radiotherapy and was reported to be alive on palliative treatment. Khor et al. [10] reported a case of NPC with an isolated brain metastasis that appeared 45 months after completion of treatment, which included chemotherapy, external radiation, and brachytherapy. The brain lesion was assumed to be a slow infection of the mastoid air cells and thus was completely excised by craniotomy. The patient was treated with whole-brain radiotherapy (total dose of 30 Gy in 10 fractions). This case is unique in that the patient had no other sites of metastasis; moreover, the lesion was located in the temporal lobe rather than the occipital lobe, as reported previously.

Direct intracranial invasion to the skull base is not uncommon in advanced NPC and considered T4 disease; however, true brain metastases of NPC are uncommon, perhaps due to the sanctuary of the brain. Even though cases of spinal cord involvement were reported, these patients did not have synchronous brain metastases. This may imply either that metastatic spread to the brain through the CSF was not the most common route or that patients did not survive long enough to develop brain metastases. Another possible explanation is that the brain is not a favorable site for developing metastasis of NPC. It seems that, in cases of disseminated aggressive disease, metastasis in uncommon sites such as the brain may be encountered.

## Figures and Tables

**Figure 1:** A Brain MRI showed a single occipital brain lesion.

**Figure 2:** FDG-PET/CT scan performed three months after completion of chemoradiotherapy showed pathological uptakes in the left cervical lymph nodes.

**Table 1:** Brain metastasis from nasopharyngeal carcinoma.

Author/year	Gender/age	Ethnicity	Systemic metastasis*	Site in the brain	Histology from brain mets	EBV from brain mets
Khor et al./1978[10]	3 patients	?	?	?	?	?
Liaw et al. /1994 [9]	Male/69	m/p Chinese	+ bone	Bilateral occipital	Squamous cell carcinoma	—
de Bree et al. /2001 [12]	Male/65	?	+	?	?	?
de Bree et al./2001 [12]	Female/64	?	+ lung	?	?	?
Ngan et al. /2002 [8]	Male/33	Chinese	+ lung	Left occipital	Undifferentiated carcinoma	+
Özyar et al./2004 [11]	Male/41	?	—	Temporal lobe	Undifferentiated carcinoma	—
Present case	Male/56	Israeli/North African	+ lung	Occipital	Undifferentiated carcinoma	+

*at time of brain metastasis diagnosis.
